This article has been retracted.

# Integrative Analyses Identify Osteopontin, LAMB3 and ITGB1 as Critical Pro-Metastatic Genes for Lung Cancer

**DOI:** 10.1371/journal.pone.0055714

**Published:** 2013-02-18

**Authors:** Xiao-Min Wang, Jing Li, Ming-Xia Yan, Lei Liu, De-Shui Jia, Qin Geng, He-Chun Lin, Xiang-Huo He, Jin-Jun Li, Ming Yao

**Affiliations:** State Key Laboratory of Oncogenes and Related Genes, Shanghai Cancer Institute, Renji Hospital, Shanghai Jiao Tong University School of Medicine, Shanghai, China; The University of Hong Kong, China

## Abstract

**Objective:**

To explore the key regulatory genes associated with lung cancer in order to reduce its occurrence and progress through silencing these key genes.

**Methods:**

To identify the key regulatory genes involved in lung cancer, we performed a combination of gene array and bioinformatics analyses to compare gene transcription profiles in 3 monoclonal cell strains with high, medium or low metastatic abilities, which were separated from the SPC-A-1sci and SPC-A-1 cell lines by limiting dilution monoclone assay. We then analyzed those genes’ biological activities by knocking down their expression in SPC-A-1sci cells using siRNA and lenti-viral shRNA vectors, followed by determinations of the invasion and migration capabilities of the resulting cell lines in vitro as well as their potential for inducing occurrence and metastasis of lung cancer in vivo. To examine the clinical relevance of these findings, we analyzed the expression levels of the identified genes in human lung cancer tissues (n = 135) and matched adjacent normal tissues by immunohistochemical (IHC) staining.

**Results:**

Three monoclonal cell strains characterized with high, medium or low metastatic abilities were successfully selected. Gene array and bioinformatics analyses implied that osteopontin, LAMB3 and ITGB1 were key genes involved in lung cancer. Knockdown of these genes suppressed human lung cancer cell invasion and metastasis in vitro and in vivo**.** Clinical sample analyses indicated that osteopontin, LAMB3 and ITGB1 protein expression levels were higher in lung cancer patients, compared to non-cancerous adjacent tissues, and correlated with lymphatic metastasis.

**Conclusions:**

We confirmed that osteopontin, LAMB3 and ITGB1 played important roles in the occurrence and metastasis of lung cancer, thus provided important clues to understanding the molecular mechanism of metastasis and contributing to the therapeutic treatment of lung cancer.

## Introduction

Lung cancer continues to be the leading cause of cancer death in the world (^>^1 million deaths per year worldwide) [1]–[2]. Metastasis is a sign and feature of malignant lung cancer and is also the main cause of lung cancer-related death and treatment failure [3]. Though over a century of intense work has focused on investigating the metastatic process, the molecular mechanisms facilitating the progression from carcinoma in situ to metastatic carcinoma remain largely elusive. It is certain, however, that metastasis is a dynamic and progressive multi-stage process. Several distinct steps are discernible in the biological cascade of metastasis: loss of cellular adhesion, increased motility and invasiveness, entry and survival in the circulation, spread into new tissue and eventual colonization of a distant site [4]. Considerable landmark studies have determined that only certain subpopulations of a primary tumor have the invasive and metastatic potential to undergo the full metastatic process of invasion, intravasation and extravasation [5]–[6]. Emerging from these studies were two concepts fundamental to our cancer lexicon: ‘metastatic subpopulations’ and ‘metastatic inefficiency’ [7]. Thus, a study of the different gene expression profiles between metastatic subpopulations and metastatic inefficiency by gene chip technology will reveal the critical genes involved in cancer metastasis.

In our previous work, we established a highly invasive cell subline (SPC-A-1sci) and a weakly invasive cell subline (SPC-A-1) by in vivo selection in NOD/SCID mice [8]. These cell lines provided an appropriate model for studying the metastatic mechanism of lung cancer. Here, we further separated 2 monoclonal cell strains from the SPC-A-1sci cell line and a monoclonal cell strain from SPC-A-1 (the parental cell line) that characterized with high, middle or low metastatic abilities, respectively, by limiting dilution monoclone assay. We then performed gene-chip combined with bioinformatics analyses on these three strains.

According to the gene array results, we found 2277 up-regulated and 2257 down-regulated genes among the three cell strains. The bioinformatics analysis revealed more details about the significant functions, pathways, expressive tendencies and signal flows of these different genes. The resulting graph from the signal-flow model indicated key regulatory roles for SPP1 (or osteopontin), LAMB3, MAPK1, and JUN in the metastasis of the SPC-A-1sci cell line.

Previously, it has been reported that cells change their cell-cell adhesion properties, rearrange their extracellular matrix (ECM) environment, and reorganize their cytoskeletons to facilitate migration and invasion.A lot of evidences have indicated that osteopontin facilitated the attachment of cells to the ECM through binding to several types of integrins (INTs), enhanced the expression and activity of MMP-2, and promoted tumor growth and metastasis through the activation of survival pathways [9]–[13]. Laminin also promoted cell adhesion and migration by interacting with INTs [14]–[16]. Here, we verified that knock-down of osteopontin, LAMB3 and ITGB1 decreased the metastasis of the SPC-A-1sci cell line through a series of experiments both in vitro and in vivo. These findings have confirmed that osteopontin, LAMB3, and ITGB1 played important roles in the metastasis of lung cancer and offer valuable clues for the study of the metastatic mechanism of lung cancer.

## Materials and Methods

### Ethics Statement

All animal experiment protocols used in this study were approved by the Shanghai Medical Experimental Animal Care Commission at Shanghai Jiaotong University (approval ID ShCI-12-023).

### Cell Lines

The human lung adeno-carcinoma cell line SPC-A-1 was obtained from Cellular Institute of Chinese Academy of Science (Shanghai, China). This cell line was originally isolated from the surgical specimens of a Chinese man with advanced lung adeno-carcinoma by Shanghai Chest Hospital and Cellular Institute of Chinese Academy of Science in 1980 [17]. The human high metastatic lung cancer cell line SPC-A-1sci was established by Ming Yao (Shanghai Jiaotong University, Shanghai cancer institute) [8]. Both lines were cultured in DMEM medium containing 10% (v/v) fetal bovine serum at 37?C, 5% CO_2_.

### Limiting Dilution Monoclone Isolation

SPC-A-1sci cells were trypsinized and resuspended in DMEM at a concentration of 100 cells per 10 mL, of which 0.1 mL was added to each well of 96-well plates already containing 0.1 mL of 10% FBS DMEM. Two weeks later, each well was observed under a microscope, and 20 monoclonal strains of SPC-A-1sci cells were selected and propagated.

### Microarray Data Analysis

Total RNA from each cell line was harvested using Trizol reagent (Invitrogen) according to the manufacturer’s instructions. Total RNA was sent to the Shanghai Biotechnology Co., Ltd (Shanghai, China). Total RNA was hybridized onto the Affymetrix U133 plus 2.0 array (Affymetrix, Santa Clara, CA, USA) and processed according to Affymetrix technical protocols. Statistical algorithms were used in the analysis of GeneChip expression data.

### Bioinformatics Analysis

#### Gene Ontology (GO) analysis

GO analysis was applied to analyze the main functions of the differentially expressed genes according to Gene Ontology, the key functional classification of the NCBI. Generally, Fisher’s exact test and χ^2^ test were used to classify the GO category, and the false discovery rate (FDR) was calculated to correct the *P*-value, with a smaller FDR corresponding to a smaller error in judging the *P*-value. The FDR was defined as , where N_κ_refers to the number of Fisher’s test *P*-values less than the χ^2^ test *P*-values. We computed *P*-values for the GO classifications of each differentially expressed gene. Enrichment provides a measure of the significance of the function: as the enrichment increases, the corresponding function is more specific, which helps us to identify those GOs in the experiment with more concrete functional descriptions. Within each significant category, the enrichment (Re) was given by: , where n*_f_* is the number of differential genes within the particular category, *n* is the total number of genes within the same category, *N_f_* is the number of differentially expressed genes in the entire microarray, and *N* is the total number of genes in the microarray [18]–[21].

#### Go-map

The Go-map, an interaction network of the significant GOs of the differentially expressed genes, was built according to the Gene Ontology classifications to identify interactions among the significant GOs directly and systemically. This map potentially summarizes the functional interactions of the differentially expressed genes under disease conditions [22]–[24].

#### Pathway analysis

Similarly, pathway analysis was used to determine the significant pathways of the differentially expressed genes according to KEGG, Biocarta and Reatome. Again, we utilized the Fisher’s exact test and χ^2^ test to select the significant pathways, and the threshold of significance was defined by the *P*-value and FDR. The enrichment was calculated according to the equation described above [19], [21].

#### Path-Net

A Path-Net was built to directly and systemically identify interactions among the significant pathways of the differentially expressed genes according to the interactions among pathways of the KEGG database. It provided a summary of the pathway interactions of the differentially expressed genes under disease conditions and assisted in determining why a certain pathway was activated [23].

### Signal-flow

External cellular stimulus affects cellular behavior and is reflected in protein interaction and gene expression kinetics. We therefore inferred a dynamic gene regulatory network, calculated according to the fold expression of genes and their interactions in pathways. The relationships of the gene expression data were inferred using a continuous time recurrent neural network (CTRNN) as an abstract dynamic model for the gene regulatory network mediating the cellular decision to migrate upon an external stimulus. The model describes the mutual influence of genes and their stimulus response as dynamic elements, regardless of how such an interaction or stimulation is realized in concrete biological terms. The CTRNN model is generally described as , where  denotes the time constant,  denotes the external input,__ denotes the weight of gene *_j_* into gene *_i_*,  denotes the offset of gene *_j_*,  denotes sigmoid activation function, and  denotes the gene *_i_* expression value at the *_t_* time point. Using this genetic algorithm, we estimated model parameters [25].

### SiRNA Transfection

siRNA oligonucleotides with the following sequences were synthesized by company(Jima,Shanghai,China): negative control siRNA, sense: 5′-UUC UCC GAA CGU GUC ACG Utt-3′ and antisense: 5′-ACG UGA CAC GUU CGG AGA Att-3′; osteopontin siRNA, sense: 5′-CCA UUC UGA UGA AUC UGA U-3′ and antisense: 5′-AUC AGA UUC AUC AGA AUG G-3′; LAMB3 siRNA, sense: 5′- CCA UUC UGA UGA AUC UGA U-3′ and antisense: 5′-AUC AGA UUC AUC AGA AUG G-3′; ITGB1 siRNA, sense: 5′-CCA UUC UGA UGA AUC UGA U-3′ and antisense: 5′-AUC AGA UUC AUC AGA AUG G-3′. Delivery of siRNAs was achieved using LipofectAMINE 2000 reagent (Invitrogen, Burlington, ON) according to the manufacturer’s instructions. Briefly, 3×10^5^ cells/well were plated into 6-well plates, cultured overnight to achieve 50–70% confluence, then washed with DMEM without serum and antibiotics. LipofectAMINE 2000 reagent and siRNA were mixed and added to the cells at final concentrations of 5 µL/well and 2.5 µg/well, respectively, followed by incubation at 37°C for 48 h.

### Preparation of Protein Extracts

Proteins from the cultured SPC-A-1sci cell lines that received siRNA treatments were harvested and pooled from 10 wells of two 6-well plates. All protein extraction procedures were performed on ice. Briefly, cells were rinsed with cold PBS, scraped by cell scraper, then transferred to 1.5 mL tubes and lysed with 200 µL of ice-cold lysis buffer per tube. After a 40-min incubation on ice, the homogenates were centrifuged at 12,000 g for 10 min at 4°C. The supernatants were collected after centrifugation.All protein extracts were stored at −20°C.

### Western Blot Analysis

Using the total protein isolated above. SDS-PAGE (12%) gels were run and subsequently transferred onto nitrocellulose membranes at 4?C. The membranes were blocked in PBS containing 5% milk for 2 hours, followed by the addition of primary antibodies against osteopontin (1∶400), ITGB1 (1∶500), LAMB3 (1∶500), and β-actin (1∶15000) Primary antibodies were incubated overnight at 4°C, followed by incubation with appropriate HRP-conjugated secondary antibodies at room temperature for 1.5 hours. The membranes were then washed with PBST (150 mM NaCl, 10 mM Tris, pH 8.0, 0.05% Tween-20), and specific proteins were detected using the HRP system.

### Real-time Quantitative PCR Analysis

Total RNA from the cultured SPC-A-1sci cell lines that received siRNA treatments was harvested using Trizol reagent according to the manufacturer’s instructions. Reverse transcription was achieved using Reverse Transcription Reagents (Takara) and following the manufacturer’s instructions. Real-time PCR analysis was performed on a 7300 Real-Time PCR System with SDS RQ Study software (Applied Biosystems) according to the manufacturer’s instructions. cDNA templates were combined with SYBR Green premix containing Rox (Takara) to perform the quantitative PCR reactions. Primers used for quantitative PCR were as follows: osteopontin forward: 5′-GACAGCCAGGACTCCATT-3′; osteopontin reverse: 5′-GATGTCAGGTCTGCGAAA -3′; LAMB3 forward: 5′-AGGCAAGAACTGTGAGCG-3′; LAMB3 reverse: 5′-GGGTTGGCGTAGGTGAGT-3′; ITGB1 forward: 5′-AATGTAACCAACCGTAGC-3′; ITGB1 reverse: 5′-CAGGTCCATAAGGTAGTAGA-3′; β-actin forward: 5′-AGTGTGACGTGGACATCCGCAAAG-3′; β-actin reverse: 5′-ATCCACATCTGCTGGAAGGTGGAC-3′. Gene expression was normalized to β-actin. All reactions were run in triplicate.

### Scratch-wound Healing Assay

The scratch-would healing assay was performed with slight modification from that previously described [26]. Cells were cultured to approximately 90% confluence in 24-well plates then starved in low serum medium (1% FBS in DMEM) overnight. A straight scratch in the cell monolayer was made using a 200 µl pipette tip to simulate a wound. The cells were rinsed with PBS and cultured with 1% FBS in DMEM for another 24 h. Three images per well were then collected from random fields using a CKX41 microscope (Olympus, Japan). The percentage of wounded area that was filled was calculated as follows: {(mean wounded breadth - mean remaining breadth)/mean wounded breadth}×100 (%).

### Migration and Invasion Assays

Cell migration and invasion assays were performed using 6.5-mm trans-well chambers (8 µm pore size, Corning) as described previously, with some modifications [27]. Cells were seeded at 100,000 cells per well into trans-well chambers and Matrigel-coated trans-well chambers for migration and invasion assays. The wells were washed with PBS after 24 h for both assays. The cells that had migrated and invaded to the basal side of the membrane were fixed and stained with H&E or crystal violet, visualized and photographed with a CKX41 microscope at 400× magnification and a DP20 Imaging system (Olympus, Japan). Images of three random fields from three replicate wells were obtained, and the number of cells that had migrated and invaded was counted.

### ShRNA Experiments

The lenti-viral shRNA vector was constructed as described previously [28]. Briefly, negative control, osteopontin, LAMB3 and ITGB1 shRNA were subcloned into the *Mlu*I/*Cla*I sites of the pLVTHM vector (Addgene) using the following oligonucleotides: 5′-CGCGTCGTAGCGACTAAACACATCAATTttc aagagaAATTGATGTGTTTAGTCGCTATTTTTTGGAAT-3′ and 5′-CGATTCCAAAAAATAGCGACTAAACACATCAATTtctcttgaaAATTGATGTGTTTAGTCGCTACGA-3′ for the negative control, 5′-CGTCGGCCATGACCACATGGACGATTTT*CAAGAG*AAATCGTCCATGTGGTCATGGCTTTTTTGGAAT-3′ and 5′-CGATTCCAAAAAAGCCATGACCACATGGACGATTT*CTCTTG*AAAATCGTCCATGTGGTCATGGCCGA-3′ for osteopontin, 5′- CGCGTCGCCCGGATCCTAGATGCAAAGA*TTCAAGAGA*TCTTTGCATCTAGGATCCGGGTTTTTTGGAAT-3′ and 5′- CGATTCCAAAAAACCCGGATCCTAGATGCAAAGA*TCTCTTGAA*TCTTTGCATCTAGGATCCGGGCGA-3′ for LAMB3 and 5′-CGCGTCGGTGTACAGATCCGAAGTTTCAT*TCAAGAG*ATGAAACTTCGGATCTGTACACTTTTTTGGAAT-3′ and 5′- CGATTCCAAAAAAGTGTACAGATCCGAAGTTTCAT*CTCTTGA*ATGAAACTTCGGATCTGTACACCGA -3′ for ITGB1. Lenti-virus generation and infection of SPC-A-1sci cells were performed as described above.

### Animal Experiments

Five- to six-week-old male nude mice were maintained under specific pathogen-free (SPF) conditions. Mice were manipulated and housed according to protocols approved by the Shanghai Medical Experimental Animal Care Commission. To analyze the in vivo metastatic capabilities of the SPC-A-1sci cells with knocked-out osteopontin, Laminin β3 or Integrin β1, 2.0×10^6^ SPC-A-1sci cells were injected into the tail veins of nude mice. Ten weeks later, all mice were sacrificed, and the lungs were removed and processed for standard histological studies by fixation in 10% formalin. The fixed samples were embedded in paraffin, and three non-sequential serial sections were obtained per animal. The sections were stained with H&E and analyzed for the presence of metastases.

### Human NSCLC Tissues

Patient samples in this study were obtained following informed consent, according to an established protocol approved by the Ethics Committee of the Shanghai Jiao-Tong University School. The data did not contain any information that may lead to the identification of the patients. Matched pairs (n = 135) of lung cancer tissues and adjacent noncancerous tissues were used for the construction of a tissue microarray (Shanghai Biochip Co., Ltd. Shanghai, China) as previously described (34). Immunohistochemical staining was performed to detect the expression of osteopontin, LAMB3, and ITGB1 in the lung cancer tissues and matched non-cancerous tissues. The primary antibodies against osteopontin, LAMB3, and ITGB1 were obtained from Sigma (1∶250), Santa Cruz (1∶50), and Abgent (1∶50). Scoring was measured by the percentage of positive cells with the following staining intensities: less than 5% scored “0”; 5–24% scored “1”; 25–49% scored “2”; 50–74% scored “3”; and more than 74% scored “4”.

### Statistical Analysis

The results are presented as the mean ± SD. Comparisons of quantitative data were analyzed by Student’s *t-*test between two groups (two-tailed; *P*<0.05 was considered significant). Fisher’s exact test was used to compare qualitative variables. Analyses were performed with SAS 9.0 for Windows.

## Results

### Different Strains of the SPC-A-1sci Cell Line Display Different Metastatic Potentials

In our previous work, a highly metastatic lung cancer cell line (named SPC-A-1sci) was established from the poorly metastatic human lung cancer cell line SPC-A-1 through three cycles of in vivo selection. The significantly higher metastatic potential of the SPC-A-1sci cell line relative to the SPC-A-1 line has been proven by a series of experiments in vivo and in vitro. To explore the causes of the high metastatic potential of cell line SPC-A-1sci, we further obtained the monoclonal cell strains SPC-A-1sci H and SPC-A-1sci M from the SPC-A-1sci cells and the monoclonal SPC-A-1L cell strain from the SPC-A-1 cell line by limiting dilution clonal assay, as described previously, with slight modifications (Figure 1A).

**Figure 1:** Different strains of the SPC-A-1sci cell line display different metastatic potentials. (A) Morphology of five monoclonal cell strains selected from the SPC-A-1sci and SPC-A-1 cell lines by limiting dilution assay. The parental SPC-A-1sci cells and SPC-A-1sci H and SPC-A-1sci M cell strains all exhibit spin shape. (B) Motility activities of SPC-A1sci, SPC-A1sci H, SPC-A1sci M, SPC-A-1 and SPC-A1 L cells were determined by scratch-wound healing assays. (C) Invasion assays of SPC-A-1sci, SPC-A1sci H, SPC-A1sci M, SPC-A-1 and SPC-A1 L cells (400× magnification). (D) Migration assays of SPC-A-1sci, SPC-A1sci H, SPC-A1sci M, SPC-A-1 and SPC-A1L cells (400× magnification). Three independent experiments were performed; results are expressed as the mean+SD; *P<0.05, **P<0.01, ***P<0.001.

To explore the metastatic potentials of SPC-A-1sciH, SPC-A-1sciM and SPC-A-1L, scratch-wound healing (Figure 1B) and migration and invasion assays were performed (Figure 1C, D). The results showed that the three monoclonal cell strains presented markedly different metastatic potentials; SPC-A-1sci H had a metastatic potential resembling that of SPC-A-1sci, SPC-A- L had a metastatic potential similar to SPC-A-1, and SPC-A-1sciM had an intermediate metastatic potential.

### Bioinformatic Analyses of Monoclonal Cell Strains with High, Middle and Low Metastatic Potentials

First, we identified genes differentially expressed by at least twofold in SPC-A-1sciH, SPC-A-1sciM cells respectively compared to SPC-A-1L cells. We found that a total of 4534 genes were differentially expressed as the intersection of SPC-A-1sciH vs. SPC-A-1L and SPC-A-1sciM vs. SPC-A-1L. Of these genes, 2277 genes were upregulated, and 2257 genes were downregulated.

To more precisely identify the key genes related to lung cancer metastasis, bioinformatic analysis was applied to analyze the functional and pathway differences between SPC-A-1sciM vs SPC-A-1L and SPC-A-1sciH vs SPC-A-1L, respectively (Figures S1, S2). The results presented in the Go-map revealed the interactions and attributions for the significant functions of the differentially expressed genes. With a threshold *P*-value <0.0001, from the functional analysis of the up-regulated differentially expressed genes, we found that significant functions were mainly associated with hemidesmosome assembly, positive regulation of erythrocyte differentiation, vesicle organization, synaptogenesis, microtubule and cytoskeleton organization and regulation, cell cycle arrest and regulation, cell adhesion and endocytosis, DNA transcription, inactivation of MAPK activity, protein amino acid dephosphorylation and intracellular protein transport. Cellular proliferation, differentiation and apoptosis were also influenced, accompanied by corresponding immune response and inflammation functions. At the same time, the majority of the down-regulated differentially expressed genes had functions in cell proliferation including: DNA replication and regulation during mitosis, spindle organization, centrosome duplication and cell-cycle checkpoint, nucleotide and negative regulation of epithelial cell proliferation as well as response to DNA damage stimulus through DNA repair and recombination, chromatin assembly or disassembly, carbohydrate, lipid and amino acid metabolism and others.

From the pathway analysis and Path-Net, we came to the conclusion that the up-regulated genes mainly participate in the MAPK signaling pathway, Wnt signaling pathway, JAK-STAT signaling pathway, TGF-beta signaling pathway, and cell adhesion. Identified genes also influence the ability of the cell to change its cytoskeleton and polarity and are involved in the occurrence, migration and metabolism of tumors. Meanwhile, the down-regulated genes mainly participated in mismatch repair and homologous recombination or were associated with the PPAR, TGF-beta, and p53 signaling pathways, ECM-receptor interactions and numerous metabolic pathways (threshold *P*-value <0.001) (Figures S3, S4).

According to the significant pathways identified above and the interactions of the differentially expressed genes involved in the pathways (according to the KEGG database), a signal-flow model was built. A quantitative regulation network, it is calculated by a neural network using the signal intensities of the differentially expressed genes. Determined from the weight difference between 2 genes and the genes that each gene is connected with, the status of SPP1, LAMB3, MAPK1 and JUN as key regulators was demonstrated (Figure 2). The expression levels of osteopontin, LAMB3, and ITGB1 were measured by qRT-PCR, and the results were concordant with the gene expression profiles. The expression levels of osteopontin, LAMB3, and ITGB1 were higher in the SPC-A-1sci H and SPC-A-1sci M cell lines than in the SPC-A-1 L cell line (Figure S5).

**Figure 2:** Bioinformatic analysis of monoclonal cell strains with high, middle and low metastatic potentials. Signal-flow model of the differential gene expression union. The dot represents the gene and the direction of the line represents the direction of the regulation. The number on the line is the regulation weight: the bigger the weight, the thicker the line and the stronger the regulatory ability. The arrow target shape of the line represents the activation regulation mode.

### SPC-A-1sci Cells Transfected with SiRNA Against Osteopontin, LAMB3, and ITGB1 Display Low Migration and Invasion In Vitro

To explore the roles of osteopontin, LAMB3 and ITGB1 in the metastasis of lung cancer, we transfected SPC-A-1sci cells with siRNA-osteopontin, siRNA-LAMB3 or siRNA-ITGB1 and performed migration and invasion assays. RT-PCR and Western blot analysis demonstrated effective knock-down of osteopontin, LAMB3, and ITGB1 in the SPC-A-1sci cells (Figure 3A, B). SPC-A-1sci cells transfected with either siRNA-osteopontin, siRNA-LAMB3 or siRNA-ITGB1 displayed significantly lower migration and invasion capabilities when compared with the parental cell line SPC-A-1 sci (Figure 3C, D). Next, osteopontin mRNA and protein expression levels were measured in SPC-A-1sci which transfected with siRNA against LAMB3 and ITGB1, the results showed knock-down of LAMB3 and ITGB1 expression levels had no influence on OPN protein expression. LAMB3 and ITGB1 had the same results (Figures S6A, B). To determine the relationship among osteopontin, LAMB3 and ITGB1,we transfected SPC-A-1sci cells with siRNA-osteopontin+siRNA-LAMB3,siRNA-osteopontin+siRNA-ITGB1,siRNA-ITGB1+ siRNA-LAMB3 and siRNA-osteopontin+siRNA-LAMB3+ siRNA-ITGB1, The migration and invasion ability of these cells co-transfected with two or more siRNA were significantly decreased compared with the invasion and migration ability of the cells co-transfected with one siRNA((Figures S6 C, D, E). The results indicate a trans-regulation role of osteopontin, LAMB3 and ITGB1 in lung cancer metastasis.

**Figure 3:** SPC-A-1 sci cells transfected with siRNA-osteopontin, LAMB3 and ITGB1 display low migration and invasion in vitro. (A) RT-PCR was performed and showed effective knock-down of expression mediated by siRNA-osteopontin, siRNA-LAMB3 and siRNA-ITGB1. (B) Western blot showed decreased expression of osteopontin, LAMB3 and ITGB1. (C and D) Migration and invasion assays of SPC-A-1sci, SPC-A1sci/siRNA-osteopontin, SPC-A-1sci/siRNA-LAMB3 and SPC-A1sci/siRNA-ITGB1 (400× magnification). Three independent experiments were performed; results are expressed as the mean +SD; *P<0.05, **P<0.01, ***P<0.001.

### Knock-down of Osteopontin, LAMB3, and ITGB1 In SPC-A-1sci Cells Resulted In Low Metastatic Potential In vivo

To further unveil whether osteopontin, LAMB3 and ITGB1 are involved in the metastasis of lung cancer in vivo,4 to 6-week-old female nude mice were randomnly divided into 4 groups and received tail vein injection of 2×10^6^ SPC-A-1sci cells transfected with the shRNA-negative control, shRNA-osteopontin, shRNA-LAMB3 or shRNA-ITGB1. Ten weeks later, lungs were collected for immunohistochemical analysis (Figure 4).

**Figure 4:** The knockdown of osteopontin, LAMB3 and ITGB1 in SPC-A-1 sci cells inhibits metastasis in vivo. Representative histological images of mouse lungs inspected for the presence of microscopic lesions (20×, upper; 400×, lower) ten weeks after tail-vein injections with SPC-A-1sci cells stably expressing shRNAs against the negative control (shRNA-NC, left 1), osteopontin (shRNA-osteopontin; left 2), Laminin β3 (shRNA-LAMB3, right 2), and Integrin β1 (shRNA-ITGB1, right 1).

We also counted the mice with lung cancer metastases and metastatic nodes in every group. As displayed in Table 1, few lung nodal metastases were detected in the mice injected with SPC-A-1sci cells transfected with shRNA-osteopontin, shRNA-LAMB3 or shRNA-ITGB1. In contrast, lung metastases were apparent in mice injected with negative control cells. Therefore, it is apparent that osteopontin, LAMB3 and ITGB1 play important roles in the metastatic process of the lung cancer cell line SPC-A-1sci.

**Table 1:** SPC-A-1sci cells transfected with shRNA against osteopontin, LAMB3 or ITGB1 resulted in less occurrence of cancer in nude mice and less metastatic nodes in lung cancer when compared to negative control.

Group	Micrometastasis(node number)	Macrometastasis(mouse number)	Metastasis(percentage)	Period(weeks)
negative control	45	6/6	100	10
shRNA-Osteopontin	11	4/6	66.6	10
shRNA-LAMB3	4	3/6	50	10
shRNA-ITGB1	8	2/6	33.3	10

### Osteopontin, LAMB3 and ITGB1 Expression Levels in Lung Cancer Are Associated with Advanced Clinical Stage, Histological Grade, and Lymph Node Metastasis

To validate the effects of osteopontin, LAMB3 and ITGB1 expression in lung cancer, we compared their expression levels in human lung cancer tissues (n = 135) and matched adjacent normal tissues by immunohistochemical (IHC) staining. Correlations between the osteopontin, LAMB3 and ITGB1 expression levels and clinicopathological characteristics of lung cancer are summarized in Table 2 and Figure 5. We found that the expression levels of osteopontin, LAMB3 and ITGB1 were significantly associated with lymph node metastasis, as these levels were significantly higher in lung cancer patients with lymphatic metastasis than in those without lymphatic metastasis. In addition, the high osteopontin and LAMB3 levels correlated positively with poor tumor differentiation, and the expression levels of osteopontin and LAMB3 were higher in the patients with advanced clinical stage than in those with early-stage lung cancer. Osteopontin, LAMB3, and ITGB1 levels were higher in primary cancers than in the adjacent controls. Overall, with respect to clinicopathological features, we found that high levels of osteopontin, LAMB3, and ITGB1 positively correlate with clinical stage, histological grade, and lymphatic metastasis in lung cancer patients, indicating that these 3 genes play important roles in lung cancer progression.

**Figure 5:** Osteopontin, LAMB3 and ITGB1 expression in lung cancer was associated with advanced clinical stage, histological grade, and lymph node metastasis. Immunohistochemical staining of osteopontin, LAMB3 and ITGB1 in lung cancer tissues and paired adjacent noncancerous tissues. The staining was scored.Scoring was measured by the percentage of positive cells with the following staining intensities: less than 5% scored “0”; 5–24% scored “1”; 25–49% scored “2”; 50–74% scored “3”; and more than 74% scored “4”.

**Table 2:** Correlation Between Osteopontin, LAMB3, ITGB1 Levels in Lung cancer Patients and Their Clinicopathologic Characteristics.

Variable	N	Osteopontin Levels (n)				LAMB3 Levels (n)				ITGB1 Levels(n)			
		0,1	2	3,4	P	0,1	2	3,4	P	0,1	2	3,4	P
Gender													
Male	81	20	14	47		35	21	25		33	24	24	
Female	35	12	9	14	0.0305*	11	16	8	0.8202	12	9	14	0.3263
Age													
□60	62	12	8	42		27	18	17		25	19	18	
>60	71	15	11	45	0.6637	31	20	20	0.965	27	16	18	0.3956
Tumorsize (cm)													
<3.5	39	8	5	26		15	13	11		18	9	12	
3.5–5	61	11	10	40	0.6461	29	12	20	0.6159	22	15	24	0.428
>5	35	9	4	22		14	14	7		12	11	12	
Histological grade													
Ι/Ι- Π	23	8	2	13		12	7	4		12	5	6	
Π	54	7	7	40	0.0156*	19	19	16	0.0153*	14	16	24	0.1931
Π-III/III	27	1	5	21		7	7	13		8	9	10	
Clinical Stage													
1AB	21	9	2	10		17	2	2		12	4	5	
2AB	16	7	2	7	<0.001*	11	1	4	<0.001*	10	1	5	0.0841
2–3AB	68	7	7	54		18	25	25		19	24	25	
3AB	5	0	1	4		0	2	3		3	1	1	
Lymphatic metastasis													
Absent	50	20	8	22		34	11	5		27	9	14	
Present	85	8	11	66	<0.001*	24	28	33	<0.001*	25	26	34	0.0174*
Carcinoma													
Primary	135	28	19	88		58	39	38		52	35	48	
Adjacent	135	68	44	23	<0.001*	114	13	8	<0.001*	95	23	17	<0.001*

P value represents the probability from a chi-square test for tissue Osteopontin, LAMB3, ITGB1 levels between variable subgroups,

* P<0.05.

## Discussion

Cancer metastasis is a continual, dynamic, complex, multi-step progression with multiple interacting factors that is one of the most important causes of cancer-related death and therapeutic treatment failure. Although confusion and perplexity exist in this field, understanding metastatic progression is significant to inhibiting the development of cancer and key to curing it.

The research in our laboratory has focused on lung cancer metastasis, and we have successfully established a highly node-metastatic mouse model of human lung cancer and obtained a human lung cancer cell line with high metastatic potential that offers us an excellent tool and platform for further research. Recently, increasing evidence has shown that in a primary malignant tumor, there exist only a few highly metastatic cells capable of metastasis and expressing the metastatic phenotype, rather than all of the tumor cells being able to invade and migrate [29], [30]. Therefore, we further separated 3 monoclonal cell strains with high, medium and low metastatic potentials from the highly metastatic heterogeneous cell line SPC-A-1sci, which has been shown to possess certain extracellular matrix transformation (EMT) characteristics [8] ^.^ We then performed a combination of gene array and bioinformatics analyses to explore the key genes involved in lung adenocarcinoma metastasis, hoping that new thoughts and clues would be indicated for the research of cancer metastasis. The study of the identified pathways, activities and functions could possibly lead to a cure for cancer.

A great deal of evidence has shown that a high level of osteopontin expression is associated with highly metastatic cancer cells [31]. Furthermore, clinical studies have manifested that osteopontin expression correlates with tumor progression and poor prognoses for patients with lung cancer. Donati et al. indicated that osteopontin expression is a significant unfavorable prognostic factor for patients with stage I NSCLC [32]. Hu et al. reported that osteopontin expression is associated with tumor growth, tumor staging, and lymph node invasion of patients with NSCLC [33]. Recently, additional studies revealed that osteopontin elevates cell migration via interaction with the ανβ3 integrin in human lung cancer cells (A549) [34]. Likewise, osteopontin is involved in tumor growth and angiogenesis of lung cancer by up-regulating vascular endothelial cell migration and proliferation via interacting with the ανβ3 integrin [35]. However, the precise biological effect of osteopontin in human lung cancer has not yet been well defined.

Laminins are a family of large glycoproteins present in various types of BM [36]. Of the many laminin isoforms, laminin-332 (laminin-5) is distinctive in both structure and behavior. Consisting of laminin α3, β3 and γ2 chains, the β3 and γ2 chains are found only in laminin-332. Laminin-332 has been related to tumor invasiveness in various types of cancer [37]–[39], and an increased expression of laminin-332 is considered a poor prognostic factor. LAMB3 enhances cell migration and tumorigenicity in SCID mice, and in collaboration with its ligand, α6β4-integrin, promotes tumorigenesis in human keratinocytes [40]. Recent evidence has also stressed the importance of β3 in prostate cancer by showing that hepsin induces cleavage of the β3 chain in prostate cancer cells, resulting in elevated [41].

In conclusion, it has become evident that osteopontin, Laminin and Integrin are associated with tumor metastasis and can enhance the migration and invasion of malignant metastatic cells from the primary tumor, mainly through changing adhesion in extracellular matrix. Here, we also provide evidence that osteopontin, LAMB3 and ITGB1 play important roles in regulating the metastatic progression of lung adenocarcinoma. Silencing the expression of each of these genes decreases the migration, invasion and wound-healing abilities of SPC-A-1 sci cells in vitro and suppresses murine lung cancer growth and metastasis in vivo. Furthermore, these 3 genes interact with each other; osteopontin and LAMB3 can both bind to ITGB1, receptors for cellular adhesion to the extracellular matrix and affect adhesion in the microenvironment to enhance the migration and invasion of highly metastatic cells. The growth and development of cancer can be inhibited if the key factors and pathways regulating the progression of cancer metastasis are discovered and blocked using the apposite antagonists. In our experiments, when we inhibit both mRNA and protein expression of osteopontin, LAMB3 and ITGB1 by applying siRNA and shRNA, the growth and metastasis of murine lung cancer decreased in vivo. Furthermore, osteopontin, LAMB3 and ITGB1 expression levels in human lung cancer tissues and matched adjacent normal tissues were examined. There was a significant association between osteopontin, LAMB3 and ITGB1 expression level that positively correlated with lymphatic metastasis in lung cancer patients.

Recent preclinical studies have identified the laminin-binding integrin α3β1 as an appealing anti-cancer target [42]. Our analysis supports the notion that gene expression differences are a crucial factor in identifying the malignant invasive cells in metastasis. Our findings, although preliminary, reveal that the knockdown of certain genes decrease the progression of lung cancer, thereby providing clues to further understand the molecular mechanism of metastasis and contribute to the therapeutic treatment of lung cancer.

## Supporting Information

Figure S1 **Go-map for SPC-A-1sciM/SPC-A-1L.** A red node indicates the function exists in the up-regulated genes; a blue node indicates the function exists in the down-regulated genes; a yellow node indicates that both the up- and down-regulated genes have the function. The direction of the arrow represents the attribution of the function.
(TIF)

Figure S2 **Go-map for SPC-A-1sciH/SPC-A-1L.** A red node indicates the function exists in the up-regulated genes; a blue node indicates the function exists in the down-regulated genes; a yellow node indicates that both the up- and down-regulated genes have the function. The direction of the arrow represents the attribution of the function.
(TIF)

Figure S3 **Path-Net for SPC-A-1sciH/SPC-A-1L.** A red node represents a pathway of the up-regulated genes; a blue node represents a pathway of the down-regulated genes; a yellow node indicates that both the up- and down-regulated genes have the pathway. An arrow represents activation and a T shape represents inhibition.
(TIF)

Figure S4 **Path-Net for SPC-A-1sciM/SPC-A-1L.** A red node represents a pathway of the up-regulated genes; a blue node represents a pathway of the down-regulated genes; a yellow node indicates that both the up- and down-regulated genes have the pathway. An arrow represents activation and a T shape represents inhibition.
(TIF)

Figure S5 **The osteopontin, LAMB3 and ITGB1 mRNA levels were determined by real-time PCR analysis in the SPC-A-1sci H, SPC-A-1sci M and SPC-A-1L cell lines.β-actin served as an internal control.**
(TIF)

Figure S6 **SPC-A-1sci cells co-transfected with two or more siRNA display low migration and invasion in vitro.** (A, B) RT-PCR and Western blot were performed and showed the expression of osteopontin, LAMB3 and ITGB1. (C and D, E) Migration and invasion assays of SPC-A-1sci co-transfected with two or more siRNA (400× magnification),sh-O+sh-L represented sh-osteopontin+sh-LAMB3, sh-O+sh-I represented sh-osteopontin +sh-ITGB1, sh-I+sh-L represented sh-ITGB1+sh-LAMB3, sh-O+sh-L+sh-I represented sh-osteopontin +sh-LAMB3+ sh-ITGB1.Three independent experiments were performed; results are expressed as the mean +SD; *P<0.05, **P<0.01, ***P<0.001.
(TIF)
